# Risk Prediction Method of Obstetric Nursing Based on Data Mining

This article has been retracted.

**DOI:** 10.1155/2022/5100860

**Published:** 2022-08-24

**Authors:** Deyan Jin

**Affiliations:** Obstetrics and Gynecology Department, Peking Union Medical College Hospital, Beijing 100730, China

## Abstract

Obstetric nursing is not only complex but also prone to risks, which can have adverse effects on hospitals. Improper handling of existing risks in obstetric care can lead to enormous harm to patients and families. Therefore, it is necessary to pay attention to the risks of obstetric nursing, especially to predict the risks in a timely manner, and take effective measures to prevent them in time, so as to achieve the purpose of allowing patients to recover as soon as possible. Data mining has powerful forecasting function, so this paper proposes to combine the data-mining-based support vector machine method and XGBoost method into a forecasting model, which overcomes the shortcomings of unstable forecasting and low accuracy of a single forecasting model. The experimental results of this paper have shown that the prediction accuracy of the SVM-XGBoost combined prediction model has reached 100%, the accuracy of the single SVM prediction model is about 78%, and the accuracy of the single XGBoost prediction model is about 75%. Compared with the single SVM model and the XGBoost prediction model, the accuracy rate had increased by about 22% and 25%, and the precision rate and recall rate are also improved. Therefore, it is very suitable to use the SVM-XGBoost combined prediction model to predict the risk of obstetric nursing.

## 1. Introduction

In order to enable obstetric nurses to learn the ability to prevent and respond to risk factors and reduce risk hazards as much as possible, managers must often implement education and training aimed at enhancing awareness of prevention and manage them in strict accordance with relevant regulations and laws. Nursing staff should also continuously strengthen risk awareness, constantly learn and generalize, strictly implement various rules and regulations, and protect the safety and health of themselves and patients. Nursing quality is an important part of hospital quality, and nursing risk prediction is a set of prediction models that reflect the impact of nursing behavior on patients. The quality of obstetric medical care is not only related to the health and safety of mothers and babies, but also related to the society's trust in the hospital. The development trend of contemporary obstetrics and gynecology nursing in order to adapt to the transformation of the medical model and the development of society, as well as the changes in people's needs for fertility, health, and medical care, the nursing model of obstetrics and gynecology is bound to adjust accordingly with the development trend of modern nursing.

The arrival of the era of big data and the rapid development of data mining have pushed China's obstetric nursing to a new level. China's obstetric nursing risk prevention platform will generate and store tens of millions of information data at all times. Using these data combined with data mining technology, we established a mathematical model to achieve efficient and complete early screening intervention for obstetric nursing risks, which has very important practical significance for preventing the occurrence of risks. The main methods of obstetric nursing risk prediction are the prediction method based on neural network algorithm and the prediction method based on decision tree algorithm. Among them, the most commonly used prediction method is based on data mining, which not only improves the prediction effect of obstetric nursing risk, but also meets the actual needs of medical examination. The innovation of this paper is that it is no longer limited to a single forecasting model in traditional data mining, but tries to combine two models to improve the forecasting accuracy of a single forecasting model. And it is proved by experiments that the prediction accuracy, accuracy of the proposed SVM-XGBoost combined prediction model, is higher than the single prediction model.

## 2. Related Work

With the increase of population, the proportion of puerperium is getting higher and higher, in order to make the puerpera have a smooth delivery and early recovery, obstetric care has become very important. O'Kelly A C discovered that preconception care through obstetric care is necessary to optimize maternal and fetal health. Maternal mortality is increasing, mainly due to the increased burden of cardiovascular disease during pregnancy, and comprehensive obstetric care is an effective way to ensure women prevent future cardiovascular complications [1]. Agatisa P K found that with advances in prenatal genetics, an important question is how to construct a patient-centered dialogue that effectively prepares pregnant women to make informed choices for screening for different genetic conditions. Compared with traditional screening, participants favored obtaining more genetic information about the fetus [2]. Ozumba has argued that although pregnancy and childbirth are considered physiological processes, the potential for catastrophic complications is very high and can develop rapidly. There is growing evidence that admission to intensive care units in high-risk patients is associated with reduced maternal mortality [3]. Keshri found people to establish obstetric care prediction methods to improve the availability of comprehensive emergency obstetric care services. To fill the gap in the shortage of obstetricians and anesthesiologists, two short-term trainings in anesthesia were carried out for serving medical staff [4]. Amosse found that distances from medical facilities and poor road infrastructure contributed to an increase in maternal deaths. His research aimed to evaluate the implementation of community-based transportation programs to improve maternal access to emergency obstetric care [5]. Scholars once believed that obstetric care is very important for pregnant women, and that effective obstetric care promotes delivery and the speed of recovery of the body. However, obstetric care also has many risks, and these risks will lead to a threat to the life of pregnant women, so it is very necessary to predict the risks of obstetric care, but scholars have not specified the method of prediction.

Data mining can not only discover the relationship between data, but also predict the risk of obstetric nursing. Hailun found that prevention and early detection of risks in obstetric care can increase the chances of successful treatment and reduce the burden. Various data mining techniques have been used for early detection of risk in obstetric care. He evaluated studies that synthesize the impact of data mining on improving risk prediction in obstetric care [6]. Tomasevic N found that the increased availability of learning data has given impetus to data mining for better prediction of obstetric care risk. His aim was to provide a comprehensive analysis and comparison of state-of-the-art supervised machine learning techniques for the task of risk prediction in obstetric care, that is, identifying “high-risk” obstetric care and predicting the probability of its future occurrence [7]. Liu Y believed that information technology in today's society is developing very rapidly, and the transmission and sharing of information has become a development trend. Data mining has gradually attracted the attention of researchers and has become a major work in the medical field. He mainly introduced data mining, aiming to provide some ideas and directions for the research of obstetric nursing risk [8]. Zhang found that the number of pregnant women whose lives are at risk due to improper obstetric nursing is huge and increasing year by year, and timely prediction of obstetric nursing risks is one of the important prevention methods. There is an urgent need to find new forecasting methods based on existing methods. He attempted to develop risk prediction models for obstetric care based on uncontrollable risk factors [9]. Scholars believe that it is a good way to use data mining in obstetric nursing risk prediction. Data mining makes the prediction accuracy rate higher, and allows relevant personnel to predict risks in advance and prevent them. But scholars have no specific experiments to prove that this method is effective.

## 3. Risk Prediction Method Based on Data Mining

As one of the outpatient departments, the obstetrics and gynecology outpatient department is mainly aimed at pregnant women and gynecological disease patients. The safety of obstetric care is currently threatened by an ageing population, weak skills, inexperience, and a lack of coordination across fields. For example, the on-duty nurse first checks the fetal position of pregnant women, if the check is improper, it will cause catastrophic consequences such as suffocation or even death of the baby and lead to nursing conflicts [10]. The increasing demand for nursing care by patients and the popularization of new technologies and equipment have put pressure on nursing staff and increased nursing risks. Nursing risk factors are shown in Figure 1:

As shown in Figure 1: nursing risks lead to death or disability of patients directly or indirectly while receiving care. Therefore, identifying, evaluating, and predicting current and potential nursing risks in order to prevent or reduce the occurrence of nursing risk events, and eliminate hidden risks and economic losses of patients are urgent problems to be solved [11]. Scientific nursing risk prediction and management can make patients have a better nursing experience and reduce the probability of risk occurrence.

### 3.1. Support Vector Machine Prediction Algorithm

In recent years, big data technology has developed rapidly and penetrated into all walks of life. How to promote the combination of medical system and big data technology is a very worthy question. The influencing factors of disease are complex and unpredictable. Therefore, this paper uses big data technology to analyze the influencing factors of disease, and uses rich physical examination data to predict disease risk, and put forward preventive measures and reasonable suggestions [12].

Prediction algorithm is an important part in the process of establishing prediction model based on data mining technology. Prediction algorithms are generally machine learning methods, and the result of the prediction target can be obtained only after the original data has been trained by the prediction algorithm to establish a model. In this paper, two prediction algorithms, support vector machine algorithm (SVM) and extreme boosting tree algorithm (XGBoost), are studied [13]. SVM is a binary classification model whose basic model is a linear classifier with the largest interval defined in the feature space.

According to the application of various methods in the current related research, support vector machine (SVM) is widely used in the field of risk prediction, and the XGBoost algorithm has performed more prominently in recent years [14]. XGBoost takes into account the situation that the training data is sparse and can specify the default direction of the branch for the missing value or the specified value, which can greatly improve the efficiency of the algorithm. Therefore, this paper explores the performance of these two data mining algorithms in obstetric nursing risk prediction, and selects a better model to apply to the construction of the integrated prediction model, as shown in Figure 2:

As shown in Figure 2: the principle of the support vector machine is derived from the perceptron. The farther the sample points are from the classification hyperplane, the more reliable the classification results are, which can also improve the generalization ability of the model and achieve the purpose of obtaining good statistical laws with a small amount of data [15]. If the dataset is linearly separable, then, let the separating hyperplane equation be :

(1) $$\begin{array}{c} w^{T}a+b=0. \end{array}$$

The distance between any point and the hyperplane is equation:

(2) $$\begin{array}{c} \gamma =\frac{\left|w^{T}+b\right|}{\left\|w\right\|}. \end{array}$$

To facilitate the computation of the transformation to w, the following relationship should be satisfied for correctly classified samples:

(3) $$\begin{array}{c} w^{T}+b\geq 1. \end{array}$$

A distance function is a functional relationship that describes the distance between two points, such as time, friction, consumption, these methods for distance measurement are gathered together, called distance function. In the support vector machine, the distance should be able to reflect the distance between the sample point and the hyperplane and the accuracy of the classification, so redefine the distance function as equation:

(4) $$\begin{array}{c} \gamma_{t}=y\left(w^{T}+b\right). \end{array}$$

According to the distance function, if *γ*_*t*_≻0, the classification is correct, otherwise the classification is wrong. But the distance function is easily affected by *w*, so the geometric distance is defined as equation:

(5) $$\begin{array}{c} \gamma {\;}^{\prime }=\frac{\gamma {\;}^{\prime }}{\left\|w\right\|}\\ =\frac{y\left(w^{T}a+b\right)}{\left\|w\right\|}. \end{array}$$

The objective function is the function of the design variables, which is a scalar. In the engineering sense, the objective function is the performance criterion of the system. The objective function of the support vector machine is transformed to maximize the geometric distance, and the support vector machine will pay more attention to the points closer to the hyperplane, and the plane parallel to the hyperplane satisfies equation:

(6) $$\begin{array}{c} y\left(w^{T}+b\right)=1. \end{array}$$

Therefore, solving the support vector machine can be transformed into solving the optimization problem of equation:

(7) $$\begin{array}{c} y=\min\frac{1}{2}\left\|w^{2}\right\|. \end{array}$$

In the mathematical optimization problem, Lagrange multiplier method is a method to find the extreme value of a multivariate function whose variables are restricted by one or more conditions. This problem can be transformed by using the Lagrange multiplier method, and then, the support vector machine can be obtained by using the optimization theory [16]. A vector machine that divides linearly separable data like this is called a linearly separable support vector machine as shown in equation:

(8) $$\begin{array}{c} s.t.y_{i}\left(w^{T}a+b\right)\geq 1-\xi_{i},\;i=1,2,\ldots ,n. \end{array}$$

Due to the nonlinearity of the data used in this paper, the kernel function should be selected for nonlinear transformation when constructing the support vector machine obstetric nursing risk prediction model [17]. In this paper, the most commonly used and effective Gaussian kernel function is used for data mapping. The definition of the Gaussian kernel function is the below equation:

(9) $$\begin{array}{c} K\left(a_{i},a_{j}\right)=\exp\left(-\gamma {\left\|a_{i}-a_{j}\right\|}^{2}\right). \end{array}$$

Gaussian kernel function, also known as radial basis (RBF) function, is a scalar function that is symmetrical along the radial direction, which is used to map finite-dimensional data to high-dimensional space. When using the Gaussian kernel function as the kernel function of the support vector machine, there are mainly two hyperparameters: the Gaussian kernel coefficient *γ* and the penalty coefficient C. Among them, *γ* represents the influence of a single sample. If the value of *γ* is small, it means that the sample has little influence on the definition of the classification hyperplane, and it is difficult to form a support vector [18].

If the value of *γ* is larger, it means that the sample has a greater influence on the definition of the classification hyperplane, and it is easier to form a support vector. The penalty coefficient C is actually the coefficient of the slack variable in the support vector machine, which is used to balance the classification error rate and the algorithm complexity, which is equivalent to the regularization coefficient. Slack variables are often introduced to facilitate solving in a larger feasible region. If it is 0, it converges to the original state, and if it is greater than zero, the constraint is relaxed, as shown in Figure 3:

As shown in Figure 3, the goal of the support vector machine is to effectively segment the feature space to obtain the best plane, and the support vector machine is determined by the support vector. The increase and decrease of non-support vectors will not affect the entire model, so the support vector machine has better stability, so redundant samples can be removed in advance, and the model efficiency can be improved. Support vector machines are good at processing high-dimensional data, and in support vector machines, the more the number of support vectors, the more complex the algorithm, and the number of generated vectors can be controlled by parameters, even if the number of dimensions is higher, it will not increase the complexity of the algorithm [19, 20].

### 3.2. XGBoost Prediction Algorithm

GBDT works well in data analysis and forecasting. It is an ensemble algorithm based on decision tree. The core of GBDT is to accumulate the results of all trees as the final result. XGBoost (algorithmic extreme gradient boosting) is an improved data mining model of GBDT, which can be used for classification and regression problems. The XGBoost regression algorithm is composed of a regression tree, and the XGBoost classification algorithm is composed of a classification tree, and the output of the classification tree is a category. In this paper, the risk of obstetric nursing is predicted, so the sample output is binary classification, and the XGBoost classification algorithm is used. The XGBoost classification algorithm is shown in Figure 4:

As shown in Figure 4, classification and regression tree (CART) is a classic decision tree that can be used to deal with classification or regression tasks involving continuous data. CART and its variants are widely used in current industrial fields. XGBoost comes from GBDT and is an improved algorithm of GBDT. GBDT only supports CART, while the base learner in XGBoost algorithm supports not only CART but also linear classifier. In addition, when XGBoost uses CART as the basic classifier, a regular term is added to the objective loss function to suppress the decline of the loss function and avoid the over-complexity and over-fitting of the model.

Parallel processing can work on different aspects of the same program at the same time. The main purpose of parallel processing is to save time for solving large and complex problems. XGBoost also adopts parallel processing in the feature dimension, and the gradient boosting decision tree in XGBoost has a sequential relationship when making decisions. Based on the current prediction of the previous round of prediction errors, each round of prediction errors is used to iteratively build a model to improve the prediction accuracy. Next, in order to understand the implementation process of the XGBoost algorithm, the loss function of XGBoost is given first, and the value of the loss function corresponding to the optimized model should be the smallest. The loss function is a function that maps the value of a random event or its related random variables to non-negative real numbers to represent the “risk” or “loss” of the random event. So, the loss function is the sum of the prediction errors of multiple trees and the regularization term, as in equation:

(10) $$\begin{array}{c} \text{obj}=\sum_{i=1}^{N}L\left(b_{i},b_{j}\right)+\sum_{m=1}^{M}\Omega \left(f_{m}\right), \end{array}$$

*b*_*j*_ represents the predicted value of sample *a*_*i*_, *b*_*i*_ represents the actual value of sample *a*_*i*_, *M* is the tree of the tree, that is, *M* iterations are performed, and *f*_*m*_ is the m^th^ tree model, that is, the m^th^ base learner. In the *f*_*m*_ expression, *J* represents the number of leaf nodes in each tree, and *J* represents the weight sum of the leaf nodes.

The generated base learner *hm* is used to fit the samples, and the best fitting value is the value that minimizes the objective loss function. The fitting process is the process of splitting the classification tree nodes, that is, selecting features and dividing them according to the different performances of the samples. Then, the optimal weight value corresponding to each leaf node can be obtained, such as equation:

(11) $$\begin{array}{c} w_{j}^{*}=-\frac{G_{i}}{H_{i}+\lambda }. \end{array}$$

The split continues until the convergence condition set by people is reached, or the number of iterations reaches the preset number of *M* times, the algorithm terminates, and the final prediction model is obtained. The XGBoost algorithm has a wide range of applications and is highly tolerant of data. Especially for sparse data, the improved gradient tree algorithm and decentralized weighting algorithm are used to ensure the accuracy of the model. In addition, the features are stored in blocks, which can be applied repeatedly during the transfer process of the tree algorithm, and the XGBoost runs very fast.

Regularization is a technique widely used in machine learning and deep learning, which can improve overfitting, reduce structural risk, and improve the generalization ability of models. Through the regularization polynomial, the regularization value is determined by the leaf node and its value. After training *k* decision trees, a sample score is predicted. The first step is to establish the model objective function. The objective function consists of two parts, as equation:

(12) $$\begin{array}{c} \text{where},\Omega \left(f\right)=\gamma T+\frac{1}{2}\lambda {\left\|w\right\|}^{2}. \end{array}$$

Taylor series is to expand a function into the form of adding power terms, the purpose is to use a relatively simple function to fit a complex function. In the second step, the pseudo-residuals are calculated to find *f* that minimizes the objective function, and the second-order Taylor expansion is used to approximate it to finally get equation:

(13) $$\begin{array}{c} {\text{Obj}}^{\left(t\right)}≅\sum_{j=1}^{n}{\left[g_{i}f_{t}\left(a_{i}\right)\right]}^{2}. \end{array}$$

Therefore, through this calculation, the objective function can be rewritten as a one-dimensional quadratic function with a leaf node score of *a*_*i*_, and the objective function can be solved.

### 3.3. Establishment of SVM-XGBoost Combined Prediction Model

A single prediction model has its own advantages and disadvantages, some models are relatively stable, but the classification accuracy is not high, and some models have high classification accuracy, but the generalization ability is not enough. Therefore, combinatorial learning can be used to integrate advantages and weaken disadvantages. Combinatorial learning is a way to make a better prediction model by integrating multiple models to form a better prediction model. In this paper, the support vector machine and the XGBoost algorithm are combined to build the model.

The determination of the kernel function is very important to the support vector machine algorithm, and SVM and its corresponding parameters will affect the structure and complexity of the high-dimensional space. The kernel function allows the support vector machine to predict high-dimensional variables well. The expression of the kernel function is as shown in equation:

(14) $$\begin{array}{c} K\left(a,z\right)=\varphi \left(a\right)•\varphi \left(z\right). \end{array}$$

In the equation, *φ* is the mapping function of the feature, and a and *z* are arbitrary features in the dataset.

The gamma value is the gamma value, which is the optimization adjustment of the curve and the auxiliary function of brightness and contrast. In the support vector machine algorithm, the gamma parameter and the penalty coefficient are the two most critical parameters. Among them, the penalty coefficient is denoted by C, and the penalty coefficient mainly deals with the situation that the prediction result is quite different from the actual result, and it is necessary to consider the promotion performance and prediction accuracy. In general, the larger the penalty coefficient, the higher the requirement for the accuracy of the prediction results. However, if the penalty coefficient is too large, it will cause overfitting, and if the penalty coefficient is too small, it will cause underfitting. The gamma parameter is brought by the radial basis kernel function, and the expression of the radial basis kernel function is as shown below:

(15) $$\begin{array}{c} K\left(a,z\right)=\exp\left(-\frac{d{\left(a,z\right)}^{2}}{2*\sigma^{2}}\right)\\ =\exp\left(-\text{ganma}\cdot d{\left(a,z\right)}^{2}\right). \end{array}$$

This paper needs to evaluate the prediction results to determine the effectiveness and superiority of the method proposed in this paper. Some common forecast evaluation criteria are described below.

Mean absolute error (MAE) is a predictive evaluation metric that uses absolute error, and then divide it by the total number of sample data to get the average absolute error. The calculation is as shown in below:

(16) $$\begin{array}{c} \text{MAE}=\frac{1}{n}\sum_{i=1}^{n}\left|b_{j}-b_{i}\right|. \end{array}$$

In which, *n* is the number of samples in the dataset, *b*_*j*_ is the predicted value, and *b* is the actual value. The mean absolute percent error (MAPE) is calculated as equation:

(17) $$\begin{array}{c} \text{MAPE}=\frac{1}{n}\sum_{i=1}^{n}\frac{\left|b_{j}-b_{i}\right|}{b_{i}}. \end{array}$$

The root mean square error (RMSE) is to calculate the square value of the absolute error of each sample data, and then, average the square value and then perform the square root operation. The calculation is as shown below:

(18) $$\begin{array}{c} \text{RMSE}=\sqrt{\frac{1}{n}\sum_{i=1}^{n}{\left(b_{j}-b_{i}\right)}^{2}}. \end{array}$$

Mean squared error (MSE) is an evaluation index that squares the absolute error between the predicted value and the actual value, and then takes the mean value. It is often used to evaluate the performance of the prediction model. The calculation is as shown below:

(19) $$\begin{array}{c} \text{MSE}=\frac{1}{n}\sum_{i=1}^{n}{\left(b_{j}-b_{i}\right)}^{2}. \end{array}$$

Comparing and analyzing the above evaluation criteria of prediction results, MAPE uses the percentage to measure the size of the deviation. MAE, MSE, and RMSE combined with the dimension of the actual value to judge the difference between the predicted value and the actual value has more practical significance. In addition, the mean square error (MSE) can also evaluate the degree of change of the sample data, and the operation is simple and the calculation speed is fast, which can greatly improve the operation efficiency.

## 4. Risk Prediction of Obstetric Nursing Based on SVM-XGBoost Combined Prediction Model

### 4.1. Prediction Effect of a Single Prediction Model

XGBoost algorithm is one of the emerging data mining algorithms in recent years. It has good application effects in various predictions, and its model parameter settings are also complicated. The parameters of XGBoost are divided into three categories: learning target parameters used to control the direction of model improvement, general parameters of the algorithm, and parameters that are further set in detail after the general parameters are determined.

The data used in this paper is a physical examination dataset from an obstetric nursing center, which records the physical index values and clinical characteristic values of patients in the obstetric nursing center. There are a total of 1000 patient nursing information data samples, as shown in Figure 5:

As shown in Figure 5, the XGBoost model has a relatively robust performance in obstetric nursing risk prediction, because when the XGBoost algorithm builds the model, each training will draw on the experience of the previous training. But this model of accumulated experience is also prone to overfitting. The SVM model performs well in obstetric nursing risk prediction, but the correction of the model is not easy to control, and it is easy to cause overcorrection.

In this paper, four indicators, recall rate, precision rate, F value, and AUC, are selected to evaluate the prediction effect of the model. Since it is hoped that the model can perform well in both recall and precision, the F-score in this model evaluation adopts the F1 value, as shown in equation below:

(20) $$\begin{array}{c} F1-\text{score}=\frac{2\times \text{recall}\times \text{precision}}{\text{recall}+\text{precision}}. \end{array}$$

The comparison table of the prediction results of the two single prediction models is shown in Table 1 and Table 2:

As shown in Tables 1 and 2: in terms of recall rate, the minimum of SVM model and XGBoost model are 0.62, and the highest are 0.67 and 0.66, respectively, only a difference of 0.01. In terms of accuracy, the minimum of SVM model and XGBoost model are 0.60 and 0.62, respectively, the highest are 0.71 and 0.70, respectively, and the highest difference is only 0.01. In terms of F1 value, the lowest values of the SVM model and the XGBoost model are 0.56 and 0.55, respectively, and the highest are 0.62 and 0.60, respectively, and the highest difference is only 0.02. In terms of AUC value, the lowest values of SVM model and XGBoost model are 0.60 and 0.61, respectively, and the highest is 0.65 in both the cases. It can be seen that the performance of support vector machine model and XGBoost model in obstetric nursing risk prediction is not much different, and the level of each index is neither high nor low, which is in a moderate level, which is not conducive to obstetric nursing risk prediction in reality.

It may be because the samples were previously sampled to balance the dataset, so the support vector would be affected by the noise at the boundary, resulting in a lower model accuracy. However, if the imbalanced data is not dealt with, the prediction results of the model may have no practical significance, so the two single prediction models perform poorly in obstetric nursing risk prediction. The prediction accuracy of the simple individual-level and complex clinical-level models is shown in Figure 6:

As shown in Figure 6: the prediction accuracy of the two models at the simple individual-level and the complex clinical-level are both below 80%, indicating that there is an overfitting phenomenon in the training process. Through the comparison of two different levels, it is found that the model at the complex clinical level considers more input variables, and the prediction accuracy of the model is slightly lower, but in general, the difference between the two levels of model accuracy is very small. From the perspective of accuracy alone, the simple individual-level model can meet the needs of daily obstetric nursing risk prediction, but in order to be more accurate, it is necessary to include more indicators at the complex clinical level for reference.

Sensitivity is used to evaluate the ability level of the model to predict patients, and Youden index is used to evaluate the total ability of the model to predict patients and non-patients. This paper compares the three major indicators of the SVM and XGBoost prediction models, as shown in Tables 3 and 4:

As shown in Tables 3 and 4: the levels of the three indicators of the two models are relatively low, and the sensitivity and specificity are below 70%, which shows that the effect of prediction and screening under this condition is not very good in the risk prediction of obstetric care. The indexes of complex clinical level were higher than those of simple individual level, which indicated that the prediction and screening effect was better and applicability was stronger in complex clinical level.

### 4.2. Prediction Effect of SVM-XGBoost Combined Prediction Model

By comparing the two different algorithms above, it is found that with the increase of input variables, the accuracy of the model is gradually improved. Therefore, only complex clinical-level predictive models are used. In order to verify the rigor of the experiment, in this paper, we conducted 5 experiments on the recall rate, precision rate, F1 value, and AUC value, as shown in Table 5:

As shown in Table 5: compared with the separate SVM and XGBoost algorithms, the three indicators of the SVM-XGBoost combined prediction model are improved. The BP-XG integrated model is better than the single prediction model in all indicators and the performance is excellent. Compared with a single prediction model, the combined prediction model of SVM-XGBoost can better handle obstetric nursing data and is more suitable as a risk prediction model for obstetric nursing.

Next, in this paper, we analyzed the MAE, MSE, and RMSE values of the SVM-XGBoost combined prediction model in 1000 samples, as shown in Figure 7:

As shown in Figure 7, the MAE, MSE, and RMSE values are all within 0.01, which fully shows that the prediction error of the SVM-XGBoost combined prediction model is less and the accuracy rate is high. The balance processing of the data will not make the prediction results fluctuate too much, and the actual prediction accuracy is high. The identification of obstetric nursing risks is accurate and comprehensive, and the comprehensive performance is relatively stable. Therefore, the XGBoost algorithm should be applied to the construction of obstetric nursing risk prediction model and should be incorporated into the risk control system of obstetric nursing.

Sensitivity, specificity, and Youden index are three important metrics when evaluating predictive models. The higher the corresponding value, the better the effect of the built model and the better the prediction performance. The three major indicators of the SVM-XGBoost combined prediction model are shown in Table 6:

As shown in Table 6: the SVM-XGBoost combined prediction model shows strong performance and the best prediction results. The sensitivity and specificity are higher than 97%, reaching the highest, the Youden index is greater than 0.95, and the misjudgment rate is only 1.12%, indicating that the learning ability and reliability of prediction through the optimization model are enhanced. The performance of the SVM-XGBoost combined prediction model is better than the other two separate algorithms, which shows that the prediction ability is greatly improved under the SVM-XGBoost combined prediction model. It can be seen that from the perspective of the three major indexes, the performance of the SVM-XGBoost combined prediction model is stronger than that of the single prediction model.

In order to verify that the SVM-XGBoost combined prediction model is suitable for obstetric nursing risk prediction, 250 samples were tested in this paper, as shown in Figure 8:

As shown in Figure 8: the accuracy rate of the training set of the SVM-XGBoost combined prediction model reaches 100%, the training effect is excellent, and the prediction optimal model is achieved. The accuracy rate of the test set also reached 90%, indicating that the SVM-XGBoost combined prediction model has strong stability and will not change greatly, so it is feasible to use it in the risk of obstetric nursing.

## 5. Conclusions

Obstetric care is one of the high-risk areas of the hospital and has a lot of responsibility. With the popularization of patients' legal knowledge and the enhancement of their awareness of rights protection, the nursing safety of obstetrics has attracted more and more attention. Strengthening obstetric nursing safety management and improving service level can reduce medical disputes. In obstetric care, there will be various risks. If the risks can be predicted on time, these risks can be effectively prevented. Therefore, this paper proposed data mining to predict the risk of obstetric nursing. Data mining can not only preprocess the data, extract effective data information, but also accurately predict the risk. Although the SVM prediction model and XGBoost prediction model proposed in this paper can also predict the risk, the accuracy rate is not so high. Experiments were conducted to prove that the SVM-XGBoost combined prediction model proposed in this paper is effective and better than the SVM prediction model and the XGBoost prediction model. The results show that the accuracy of the SVM-XGBoost combined prediction model is indeed higher than that of the single SVM prediction model and the XGBoost prediction model. Therefore, the application of data mining technology to the prediction of obstetric nursing risk is also a major discovery of the article. However, there are still many deficiencies in the article. The author will continue to consolidate professional knowledge and strive to do better.

## Figures and Tables

**Figure 1:** Nursing risk factors.

**Figure 2:** Schematic diagram of support vector machine.

**Figure 3:** Gaussian kernel function.

**Figure 4:** XGBoost classification algorithm.

**Figure 5:** Accuracy of SVM model and XGBoost algorithm (a) the accuracy of the SVM model (b) the accuracy of the XGBoost algorithm.

**Figure 6:** The prediction accuracy of the two models in different environments (a) the prediction accuracy of the two models at the simple individual-level (b) the prediction accuracy of the two models at the complex clinical-level.

**Figure 7:** Error of SVM-XGBoost combined prediction model.

**Figure 8:** The accuracy of the combined prediction model of SVM-XGBoost under the training set and test set (a) the accuracy of the model in the training set (b) the accuracy of the model in the test set.

**Table 1:** Effects of the SVM model.

Number of experiments	Recall	Accuracy	F1 value	AUC value
1	0.65	0.71	0.58	0.65
2	0.62	0.68	0.59	0.61
3	0.63	0.65	0.56	0.62
4	0.64	0.69	0.61	0.60
5	0.67	0.60	0.62	0.63

**Table 2:** Effect of XGBoost model.

Number of experiments	Recall	Accuracy	F1 value	AUC value
1	0.66	0.70	0.56	0.62
2	0.63	0.69	0.60	0.63
3	0.64	0.68	0.58	0.61
4	0.65	0.67	0.57	0.64
5	0.62	0.62	0.55	0.65

**Table 3:** SVM prediction model.

Model	Simple personal level	Complex clinical model
Sensitivity	67.49%	68.90%
Specificity	67.83%	65.36%
Misjudgment rate	25.87%	25.89%
Youden index	0.563	0.588

**Table 4:** XGBoost prediction model.

Model	Simple personal level	Complex clinical model
Sensitivity	68.43%	69.77%
Specificity	68.28%	66.65%
Misjudgment rate	26.89%	26.42%
Youden index	0.657	0.672

**Table 5:** Effect of SVM-XGBoost combined prediction model.

Number of experiments	Recall	Accuracy	F1 value	AUC value
1	0.78	0.89	0.77	0.72
2	0.80	0.87	0.78	0.75
3	0.83	0.93	0.79	0.79
4	0.87	0.92	0.82	0.84
5	0.90	0.91	0.85	0.87

**Table 6:** SVM-XGBoost combined prediction model.

Model	Simple personal level	Complex clinical model
Sensitivity	98.52%	98.81%
Specificity	97.76%	97.93%
Misjudgment rate	1.12	1.12
Youden index	0.97	0.96

## Data Availability

The datasets generated during and/or analyzed during the current study are not publicly available due to sensitivity and data use agreement.

## References

[1] O’Kelly A. C., Scott N., DeFaria Yeh D. (2021). Delivering coordinated cardio-obstetric care from preconception through postpartum. *Cardiology Clinics*.

[2] Agatisa P. K., Mercer M. B., Mitchum A., Coleridge M. B., Farrell R. M. (2018). Patient-centered obstetric care in the age of cell-free fetal DNA prenatal screening. *Journal of Patient Experience*.

[3] Ozumba B., Ajah L. O., Obi V. (2018). Pattern and outcome of obstetric admissions into the intensive care unit of a southeast Nigerian hospital. *Indian Journal of Critical Care Medicine : Peer-reviewed*.

[4] Keshri V. R., Garg B. S. (2021). Operational barriers in providing comprehensive emergency obstetric care by task shifting of medical officers in selected states of India. *Indian Journal of Community Medicine: Official Publication of Indian Association of Preventive & Social Medicine*.

[5] Amosse F., Boene H., Kinshella M. L. W. (2021). Implementation of a community transport strategy to reduce delays in seeking obstetric care in rural Mozambique. *Globalization and Health: Science and Practice*.

[6] Liang H., Yang L., Tao L. (2020). Data mining-based model and risk prediction of colorectal cancer by using secondary health data: a systematic review. *Chinese Journal of Cancer Research*.

[7] Tomasevic N., Gvozdenovic N., Vranes S. (2020). An overview and comparison of supervised data mining techniques for student exam performance prediction. *Computers & Education*.

[8] Liu Y., Yu Z., Yang Y. (2021). Diabetes risk data mining method based on electronic medical record analysis. *Journal of Healthcare Engineering*.

[9] Zhang H. . (2020). Development of a risk prediction model for central-line–associated bloodstream infection (CLABSI) in patients with continuous renal replacement therapy. *Infection Control & Hospital Epidemiology*.

[10] Chidozie Egejuru N., Olayinka Olusanya S., Onyenonachi Asinobi A., Joseph Adeyemi O., Oluwatimilehin Adebayo V., Adebayo Idowu P. (2019). Using data mining algorithms for thalassemia risk prediction. *International Journal of Biomedical Science and Engineering*.

[11] Xin W. (2018). Enterprise financial risk control in the perspective of internal control based on data mining. *IPPTA: Quarterly Journal of Indian Pulp and Paper Technical - A*.

[12] Gopinath G., Gv K. G., Sasikumar H., Tamilanban Y., Patil J., Gopinath G. (2021). A novel artificial intelligence based internet of things for fall detection of elderly care monitoring. *Journal of Intelligent Systems and Internet of Things*.

[13] Li X., Jiao H., Li D (2020). Intelligent medical heterogeneous big data set balanced clustering using deep learning. *Pattern Recognition Letters*.

[14] Zhou Z. R., Wang W. W., Li Y. (2019). In-depth mining of clinical data: the construction of clinical prediction model with R. *Annals of Translational Medicine*.

[15] Xie S., Yu Z., Lv Z. (2021). Multi-disease prediction based on deep learning: a survey. *Computer Modeling in Engineering and Sciences*.

[16] Le H. M., Tran T. D., Tran L. V. (2018). Automatic heart disease prediction using feature selection and data mining technique. *Journal of Computer Science and Cybernetics*.

[17] Humayun S., Chaudhary S., Malik N., Shamila Ijaz M. (2021). Obstetric care in COVID-19: strategy in a tertiary care setting. *Annals of King Edward Medical University Lahore Pakistan*.

[18] Salter C. L., Olaniyan A., Mendez D. D., Chang J. C. (2021). Naming silence and inadequate obstetric care as obstetric violence is a necessary step for change. *Violence Against Women*.

[19] Seid M. (2021). Utilization of parthogrph and associated factors among obstetric care providers in public health institutions. *Bu. International Journal of Current Research*.

[20] Frank Z. C., Caughey A. B. (2018). Pregnancy in women with a history of uterine rupture. *Obstetrical and Gynecological Survey*.

